The article "Research on Classification of Primary Liver Cancer Syndrome Based on Data Mining Technology" was retracted in 2023. Reasons: signs of a paper mill; compromised peer review; unreliable results or conclusions.

# Research on Classification of Primary Liver Cancer Syndrome Based on Data Mining Technology

**DOI:** 10.1155/2022/2629509

**Published:** 2022-01-07

**Authors:** Jiwei Fang, Jianfeng Li

**Affiliations:** ^1^General Practice Medicine, The First Affiliated Hospital of Nanchang University, Nanchang 330006, China; ^2^Department of General Surgery, The First Affiliated Hospital of Nanchang University, Nanchang 330006, China

## Abstract

This study is based on the analysis of the status quo of the research on liver cancer syndromes, starting with the clinical objective and true four-diagnosis information of TCM inpatients with primary liver cancer, using computer data mining technology to analyze and summarize the syndrome rules from the bottom to the top. Let the data itself show the essence of liver cancer syndrome. First, with the help of hierarchical cluster analysis, we can understand the general characteristics through the rough preliminary classification of the four-diagnosis information of liver cancer patients. Then, with the help of the emerging and mature hidden structure model analysis in recent years, through data modeling, the classification of common syndromes of liver cancer and the corresponding relationship with the four-diagnosis information are comprehensively analyzed. Finally, considering the inherent shortcomings of implicit structure and hierarchical clustering based on the assumption that there is a unique one-to-one correspondence between the four diagnostic information factors and the class (or hidden class) when classifying, we plan to use factor analysis and joint cluster analysis, as supplementary means to further explore the classification of liver cancer syndromes and the corresponding relationship with the four-diagnosis information.

## 1. Introduction

Primary liver cancer is one of the fast-progressing malignancies among various solid malignancies. Its mortality rate ranks third among male patients (after gastric cancer and esophageal cancer) and fourth among female patients. Clinically, primary liver cancer can be divided into massive type (5–10 cm), nodular type (3–5 cm), small liver cancer (3 cm), and diffuse type according to the size of the tumor. According to the pathological characteristics of tumor cells, it can be divided into thin beam type, thick beam type, clear cell type, hepatocyte-bile duct cell type, pseudoglandular tube type, dense type, sclerosis type, fiber lamellar type, giant cell type, vasodilatation type, and other types, of which the thick beam type is the majority. Before the 1960s, various detection methods were lacking, and when the clinical diagnosis was clear, it was close to the middle and late stages [1]. At that time, it was believed that the natural course of primary liver cancer was 3–6 months. Since the 1970s, the importance of AFP alpha-fetoprotein in the diagnosis of primary liver cancer has been gradually affirmed. Significant progress has been made in the early detection of liver cancer. At the same time, some people proposed the significance of small liver cancer and subclinical liver cancer, which completely changed the understanding of the natural course of primary liver cancer. The natural course from the discovery of elevated AFP to the death of liver cancer patients is about two years or longer. Since the 1980s, imaging (ultrasound CTMRI) has been rapidly developed and popularized, and there is a reliable basis for the localization and diagnosis of liver cancer, and the treatment rate and 5- to 10-year survival rate have shown a trend of increasing year by year [2, 3].

The article "Research on Classification of Primary Liver Cancer Syndrome Based on Data Mining Technology" was retracted in 2023. Reasons: signs of a paper mill; compromised peer review; unreliable results or conclusions.

However, primary liver cancer is an intractable and harmful disease, and the rate of surgical resection is low. At present, the 5-year survival rate after radical resection of liver cancer is about 30%–66.7%, and the recurrence rate after 5 years can be as high as 71%–95% [4, 5]. This has become the main factor affecting the long-term efficacy. Because the information related to this disease is too scattered and not easy to obtain comprehensively, doctors and patients can only form qualitative judgments and quantitative descriptions of the prognosis of the disease through knowledge and experience accumulation. Therefore, the problem of simple and rough qualitative judgments and poor accuracy in predicting disease prognosis has long existed, and it is difficult to convince doctors and patients. For such critical diseases, the patient spends a lot of money, and the expectation of curing the disease is high. If the doctor's prediction of the prognosis of the disease is severely distorted, it will easily lead to doctor-patient disputes. Therefore, predicting the prognosis of primary liver cancer is a challenging and socially significant subject [6].

At present, there are no mature and large sample reports on the prognosis prediction of primary liver cancer, and there are no reports on the prognosis prediction combined with clinical imaging and laboratory. Relevant clinical studies are limited to some medical statistical conclusions on the prognosis and survival of primary liver cancer. Its research methods are also limited to retrospective analysis of clinical static data with a small sample size, mainly including early detection, tumor size and distribution, envelope status, TNM staging, liver function status, radical cure classification, tissue type, degree of differentiation and portal vein tumor thrombus, and so on. Many scholars have done a lot of work in the laboratory research of predictive indicators, and found that certain oncogenes [7], tumor suppressor genes, growth factors, and other factors have a great relationship with cancer aggressiveness and poor prognosis. However, irrespective of the clinical or laboratory aspects, there is still a lack of systematic methods for predicting the prognosis of primary liver cancer, and the modeling and softwarization of methods have not been realized.

The article "Research on Classification of Primary Liver Cancer Syndrome Based on Data Mining Technology" was retracted in 2023. Reasons: signs of a paper mill; compromised peer review; unreliable results or conclusions.

Based on the above understanding, the research team intends to apply computer technology to start with the objective and true clinical information of the fourth diagnosis of traditional Chinese medicine in patients with primary liver cancer. Cluster analysis, hidden structure model analysis, factor analysis, and other data mining techniques are used to explore the characteristics of liver cancer syndromes. Basic pathogenesis of liver cancer syndromes are summarized and related research and exploration are conducted. These have important practical significance for deepening the understanding of liver cancer syndromes and guiding their clinical differentiation and treatment [8, 9].

In this paper, analysis of the status quo of the research on liver cancer syndromes is presented which is initiated with the clinical objective and true four-diagnosis information of TCM inpatients with primary liver cancer. Let the data itself show the essence of liver cancer syndrome. First, with the help of hierarchical cluster analysis, we can understand the general characteristics through a rough preliminary classification of the four-diagnosis information of liver cancer patients. Then, with the help of the emerging and mature hidden structure model analysis in recent years, through data modeling, the classification of common syndromes of liver cancer and the corresponding relationship with the four-diagnosis information are comprehensively analyzed.

The rest of the manuscript is organized as follows. Related work is presented in the following section, which is followed by a detailed discussion and explanation on the proposed methodology and its effectiveness in resolving the aforementioned issue. Experimental results were presented to justify various claims of the proposed scheme in terms of different performance evaluation metrics. Finally, the concluding remarks are given.

## 2. Related Work

The continuous development of medical testing methods in the twentieth century has provided doctors with more powerful help in diagnosing diseases, and with the rapid development of computers and related technologies, computer-aided diagnosis has also attracted more and more attention [10].

The article "Research on Classification of Primary Liver Cancer Syndrome Based on Data Mining Technology" was retracted in 2023. Reasons: signs of a paper mill; compromised peer review; unreliable results or conclusions.

With the computerization of hospitals, many hospitals began to use Picture Archiving and Communication System. These hospitals have collected a large number of patients' medical images (including SPECT, PET, MRI, HRCT, etc.) and other relevant medical parameters. The goal of a computer-aided medical diagnosis system is how to make full use of the previous confirmed cases and the doctor's diagnosis experience plus the current patient information, so that the computer can help the doctor to diagnose the disease quickly and effectively. In the past, medical-aided diagnosis systems were all expert systems based on knowledge, and they often had the following deficiencies: (1) the bottleneck of knowledge acquisition, (2) the fragility of knowledge, and (3) the monotonicity of reasoning.

The specific manifestation is that about 60%–70% of the time spent on knowledge acquisition is to develop an expert system based on rules and knowledge. The method adopted by technology is that experts express their heuristic classification experience through a series of domain rules [11–13]. Because most experts have difficulty in displaying their domain knowledge, the application effect is sometimes not ideal. And when human experts use this knowledge, they use more thinking methods such as association. In short, obtaining information and expression from experts is challenging, and it has qualitative and subjective features that are difficult to quantify and objectively represent. In order to overcome the above shortcomings, an intelligent diagnosis system similar to NNES (Neural Network Expert System) has emerged. Its advantages are: it has a learning function, large-scale parallel distributed processing [14], and a global collective role to realize automatic knowledge acquisition. Parallel association and adaptive reasoning can be realized, and the system has real-time processing capabilities and good robustness. Compared with the traditional expert system ES, this type of intelligent diagnosis system has superior performance in classification diagnosis and classification-based intelligent control and optimization solutions. But, there are some inherent shortcomings, such as: (1) more suitable for solving some small-scale problems; (2) to a large extent limited by the training data set; (3) limited to the acquisition of knowledge of common-sense problems; and (4) knowledge representation, the processing is complicated and inefficient, and there is a “black box” operation.

All these determine that the current intelligent diagnosis system cannot have a high level of intelligence [15, 16]. However, the introduction of data mining and knowledge discovery in such systems can alleviate or partially solve some of the abovementioned problems, which is also the development direction of today's intelligent diagnosis systems.

The article "Research on Classification of Primary Liver Cancer Syndrome Based on Data Mining Technology" was retracted in 2023. Reasons: signs of a paper mill; compromised peer review; unreliable results or conclusions.

Data mining is developed from machine learning, a branch of artificial intelligence, and has a history of more than ten years. Data mining is a nontrivial process of obtaining correct, novel, potentially applicable, and ultimately understandable patterns from the database. Knowledge discovery refers to the overall process of discovering useful knowledge from data. Data mining can be considered as a step in knowledge discovery. It is the core of knowledge discovery, so the two terms can be used interchangeably. It is an emerging field with broad development prospects formed by the intersection of many disciplines such as artificial intelligence, machine learning, pattern recognition, statistics, database, and knowledge base data visualization [17, 18].

The original processing object of the computer-aided medical diagnosis system is the medical information database. This object is actually a multimedia database, which may contain medical images of patients, used by doctors for diagnosis, related pathological parameters, laboratory results, diagnosis results, and related reference parameters such as age, gender, medical history, discharge/admission time, etc. In short, it is a multimedia database with text, graphics, or images, as well as numbers or data information. However, current data mining techniques are mainly applied to relational databases, transaction databases, and data warehouses based on structured data. The mining of complex types of data is still in its infancy. Complex data include complex objects, spatial data, multimedia data, time series data, text data, and web data. Therefore, it is necessary to conduct data mining and knowledge discovery on medical information databases. Discovering the rules and patterns of medical diagnosis to assist doctors in disease diagnosis is a challenging and promising task. The current data mining object-medical information database can be summarized into two categories: (1) medical imaging plus other related medical parameter database and (2) pure medical parameter database without medical imaging [19–21].

In most cases, the goal of data mining and knowledge discovery on medical databases should be to diagnose diseases or discover medical diagnosis rules based on previous experience like doctors. For example, if a breast tumor is diagnosed as benign or malignant, the MRI image data of the brain can be used to distinguish whether the patient has meningioma or an astrocytoma [22]. According to the SPECT image of the patient's heart, the myocardial perfusion is classified or diagnosed with coronary artery disease or without the disease, and the 12 types of chest pain are classified, and so on. In addition, there are also sequential time pattern discoveries, such as the discovery of time patterns in the course of HIV disease, the pattern extraction of nuclear medicine parameters, and the discovery of causal relationships among several parameters, such as the discovery of children's fracture databases and scoliosis databases. The causal relationship between pattern extraction and its medical parameters was discovered.

The article "Research on Classification of Primary Liver Cancer Syndrome Based on Data Mining Technology" was retracted in 2023. Reasons: signs of a paper mill; compromised peer review; unreliable results or conclusions.

Syndrome is the basis of TCM syndrome differentiation and treatment, and it is also the core and bottleneck problem that restricts the development of TCM. At the same time, it is one of the hot spots of TCM clinical research. It is traditionally believed that syndromes cover the symptoms and signs shown by patients that can reflect the location, nature, degree, or development trend of the disease. Academicians summarized the characteristics of TCM syndromes as “internal reality and external deficiency, dynamic time and space, multidimensional interface”, and believed that TCM syndrome is a nonlinear, multidimensional structure composed of multiple factors through different connection forms and strengths, a complex giant system that can be combined infinitely. The Qing Dynasty physician Ye Tianshi said in the “Clinical Guide to Medical Cases”: “The way of medicine cares about the identification, legislation, and prescription. These are the three key points. One is sloppy and unsatisfactory. However, among the three, identification is particularly important.” It can be seen that syndrome differentiation is the key to the success of syndrome differentiation and treatment, and the standardization of TCM syndromes is of great significance to the improvement and development of TCM clinical diagnosis and treatment, as well as the communication and exchange of TCM and Western medicine. Since the 1980s in the 20th century, China has carried out modern standardized research on TCM syndromes, and has achieved certain results. In recent years, with the increasing development and penetration of knowledge in many subjects such as mathematical statistics, information technology, epidemiology, fuzzy mathematics, etc., the research methods and models of TCM syndromes have been increasing. At present, there are still difficulties in the research method of this open and complex giant system.

Because the data of TCM syndromes have the characteristics of large amount, vagueness, randomness, and concealment, how to discover potential relationships and laws between data and how to evaluate the next development trend based on existing data has become a difficult problem for TCM researchers. Data Mining is precisely the knowledge acquisition technology that can deal with the complexity of data. It is similar to the process of TCM syndrome differentiation. It can realize the intelligent analysis of massive data. The essence of things and the implicit patterns or laws that can predict their development trend are to be obtained. Data mining technology integrates database, statistics, artificial intelligence, pattern recognition, high-performance computing, and other multidisciplinary knowledge, and its concept is equivalent to knowledge discovery in the database.

The article "Research on Classification of Primary Liver Cancer Syndrome Based on Data Mining Technology" was retracted in 2023. Reasons: signs of a paper mill; compromised peer review; unreliable results or conclusions.

## 3. Proposed Methodology

### 3.1. Research Objective

The cases investigated in this study were all from inpatients with primary liver cancer in the Department of Traditional Chinese Medicine of a hospital. A total of 650 samples of effective primary liver cancer cases were collected, including 552 males and 98 females; the age range was 25–82 years, with an average age of 50.73 ± 6.54 years; 73 cases were clinically staged in stage Ia, 24 cases in stage Ib, and there were 37 cases in stage IIa and 164 cases in stage IIb.

### 3.2. Diagnostic Criteria

The diagnosis and clinical staging standards of primary liver cancer refer to the “Clinical Diagnosis and Staging Standards of Primary Hepatocarcinoma” formulated by the Chinese Anti-Cancer Association at the National Hepatocarcinoma Academic Conference held in Guangzhou in September 2001. The diagnostic standards are the following:

1. AFP >400 ug/l, can exclude pregnancy, germline embryogenic tumors, metastatic liver cancer, and active liver disease, can palpate enlarged, hard, and large nodular masses of the liver, or can do imaging, finding patients with space-occupying lesions characteristic of liver cancer
2. AFP <400 ug/l, can exclude pregnancy, germline embryogenic tumors, metastatic liver cancer, and active liver disease, and there are two kinds of imaging examinations to find space-occupying lesions with liver cancer characteristics or there are two types of serum liver cancers and those with positive markers and a space-occupying lesion with characteristics of liver cancer can be found on an imaging examination
3. Patients with clinical manifestations of liver cancer and confirmed extrahepatic metastatic lesions (including visible bloody ascites or cancer cells found) and metastatic liver cancer can be excluded

### 3.3. Inclusion and Exclusion Criteria

Inclusion criteria: The diagnosis meets the primary liver cancer diagnosis criteria established by the National Liver Cancer Academic Conference in September 2001: those who gave informed consent to this survey.

The article "Research on Classification of Primary Liver Cancer Syndrome Based on Data Mining Technology" was retracted in 2023. Reasons: signs of a paper mill; compromised peer review; unreliable results or conclusions.

Exclusion criteria: Those who have proved to be complicated with primary diseases such as severe hematopoietic system and cardiovascular and cerebrovascular diseases; those who are critically ill and are not suitable for investigation; those who have difficulty in verbal expression; those who do not cooperate with the investigation; and those who fill in the form irregularly.

### 3.4. Statistical Analysis of the Proposed Methods

The “Traditional Chinese Medicine Liver Cancer Syndrome Questionnaire” developed based on literature retrieval, clinical practice, and expert discussions collects information on the four diagnoses of TCM inpatients with liver cancer, and strictly controls the quality of the survey. Clinical physicians conduct bedside collection. The tongue and pulse conditions are distinguished by two professionals with the title of attending physician or above at the same time, and the patient's objective tongue and pulse information is collected with the help of the tongue diagnosis information collection system and pulse meter. Make judgments of TCM syndromes and minimize selectivity and measurement bias.

The collected four-diagnosis information of TCM for 650 patients with primary liver cancer was assigned “1, 0” according to “with and without”, and entered into Microsoft Excel 2007 software. Two persons were used to enter data and conduct comparative and logical inspections. Afterwards, a person will be assigned for sampling inspection, and the sampling rate shall not be less than 30%. Combining frequency analysis, literature review, expert argumentation, and clinical epidemiological investigation, the research team finally screened out 57 four-diagnosis information data of traditional Chinese medicine, including flank pain, anorexia, fatigue, emotional depression, red tongue, and pulse string to participate in the study.

In this study, the R 3.0.1 software was used to perform systematic clustering analysis of the data using the sum of squared deviation method. The Lantern 3.1.2 software developed by the Hong Kong University of Science and Technology was used to select the EAST algorithm to analyze the hidden structure model of the data. Using the R 3.0.1 software, factor analysis and cluster analysis were performed on the data to deeply explore the symptoms and pathogenesis of primary liver cancer.

## 4. Experimental Result

### 4.1. Cluster Analysis Results

Cluster analysis is an exploratory analysis of the data. In this study, the 57 four-diagnosis information data of traditional Chinese medicine can be regarded as 57 variables. The R-type cluster in the cluster analysis can be used to classify these 57 variables. The variables with collinearity are classified into one category, the dimensionality reduction of the index is achieved, and the gradual hierarchical classification of variables is realized, thereby completing the classification of the four-diagnosis information group.

The article "Research on Classification of Primary Liver Cancer Syndrome Based on Data Mining Technology" was retracted in 2023. Reasons: signs of a paper mill; compromised peer review; unreliable results or conclusions.

In the process of clustering, 57 variables are gradually classified and merged. Each category is a group of four-diagnosis information group. The four-diagnosis information has a strong tendency to gather together and is governed by a certain specific law, that is, the basic pathogenesis law. Combining professional knowledge and clustering results, we think it is more reasonable to classify into 8 categories.

  Category 1: chest tightness, fullness of the abdomen, pain in the stomach, dizziness, chills, fullness of the stomach, and anorexia, which roughly reflect the pathogenesis of air block
  Category 2: astringent pulse, heavy head and body, and shoulder and back pain, suggesting that it may be related to stagnation of qi and blood stasis
  Category 3: pale complexion; dirty mouth; dry stool; lump under the side; spontaneous sweating; heat of the hands, feet, and heart; edema of the lower extremities; and thirst, mainly including the two factors of toxic heat and deficiency
  Category 4: pale lips and nails, pale face, oliguria, pulse count, chest pain, emotional depression, and pleural effusion, which manifests the pathogenesis characteristics of qi and blood stasis and mixed deficiency and excess.
  Category 5: fever and hot flashes are all related to fever.
  Category 6: tinnitus, weak pulse, nausea and vomiting, thin stool filter, ascites, petechiae and ecchymosis tongue, and white fur, which roughly reflects the pathogenesis of yang deficiency of the spleen and kidney.
  Category 7: frequent nocturia; hiccups and warm air; insomnia; weakness in waist and knees; yellowish body; dry mouth and throat; bitter mouth; yellow urine; flank pain; fatigue, mainly manifesting liver and kidney insufficiency; lack of righteousness deficiency; and liver and gallbladder damp-heat content.
  Category 8: yellow fur, greasy fur, purple tongue, fat large teeth marks on tongue, thin pulse, dull complexion, stringy pulse, and sublingual network.

The results of cluster analysis can reflect the clinical reality of liver cancer syndromes to a certain extent, suggesting that the pathogenesis of liver cancer is mainly solid or a mixture of deficiency and excess, and the syndrome manifestations are stagnation of qi, stagnation of qi and blood stasis, mutual accumulation of dampness and blood stasis, and deficiency of blood. Stasis, intense heat toxin, damp-heat of liver and gallbladder, deficiency of liver and kidney, and yang deficiency of spleen and kidney are common. However, due to the systematic clustering, each piece of information will only be simply classified into a certain category, so that when the clustering results are discussed based on professional knowledge, some deviations will inevitably occur, such as fatigue. Although it is more common in deficiency syndromes, such as qi deficiency, in clinical syndromes, qi stagnation, dampness, blood stasis, and other solid syndromes, patients often have similar manifestations of varying severity. From the perspective of the classification of syndromes, liver and gallbladder damp-heat and liver and kidney deficiency are grouped into the same syndrome category, which is not completely in line with clinical reality. Therefore, combining the connotation of TCM syndromes, trying more mathematical analysis methods for the classification of liver cancer syndromes, and exploring the optimal scheme is also one of the important topics of its syndrome research.

The article "Research on Classification of Primary Liver Cancer Syndrome Based on Data Mining Technology" was retracted in 2023. Reasons: signs of a paper mill; compromised peer review; unreliable results or conclusions.

### 4.2. Analysis Results of Hidden Structure Model

Latent structure model is a mathematical model developed by Professor Zhang Lianwen from the Department of Computer Science and Engineering of Hong Kong University of Science and Technology, which is specially used in the objective and quantitative research of TCM syndromes. A hidden model of a tree-like Bayesian network is used to perform hierarchical clustering, comprehensively evaluate the clinical objective of four-diagnosis information data, and reveal the hidden rules to guide the differentiation of syndromes. The model is written in JAVA language, and the heuristic double hill climbing algorithm is used for hierarchical exploration. By introducing hidden variables that cannot be directly observed but need to be obtained through comprehensive analysis, the explicit variables that can be directly observed are multidimensionally layered. Clustering establishes a hidden structure model by analyzing the relationship between hidden variables and explicit variables, and between hidden variables and hidden variables, and fully excavates the characteristics of potential hidden variables.

#### 4.2.1. The Information Curve and the Interpretation of the Pathogenesis Law

It can be seen from the analysis results that the hidden structure model includes 14 hidden variables Y0, Yl, Y2 to Y13, and each hidden variable represents a division of the data sample from a certain angle or side. The number in parentheses after each hidden variable means that the hidden variable divides the population into several hidden categories. For example, Y3 represents the number of hidden variables. Y3 is 2, which means that Y3 divides the population into 2 hidden categories. The thickness of the line between the variables in the hidden structure model reflects the strength of the correlation between the variables. For example, the hidden variable Y8 has a close relationship with fever and hot flashes, but has a weaker relationship with the pulse number, ascites, and pale nails. Through analysis, the information curve of each hidden variable can accurately grasp the main four-diagnosis information contained in each hidden variable, and then grasp the hidden pathogenesis law.

The article "Research on Classification of Primary Liver Cancer Syndrome Based on Data Mining Technology" was retracted in 2023. Reasons: signs of a paper mill; compromised peer review; unreliable results or conclusions.

The latent variable Y0 includes two pieces of information: flank pain and spontaneous sweating. The importance of Y0 is flank pain and spontaneous perspiration in order of importance. Among them, flank pain is one of the most common clinical symptoms of liver cancer. The information coverage reached nearly 90%, and it can be considered that the influence of spontaneous sweat on Y0 is very weak, so the implicit variables may be related to qi and blood stagnation.

The latent variable Y1 includes 9 information such as heavy head and sleepiness, emotional depression, full stomach and wrist fullness, stomach and wrist pain, chest pain, chest tightness, dizziness, and chills. The importance of Y1 information in descending order is fullness of stomach cyst, chills, chest tightness, pain of stomach prolapse, dizziness, and fullness of abdomen. They contain more than 95% of the information in this category, combined with professional knowledge analysis. This information group roughly reflects the pathogenesis law of Qi block.

The latent variable Y2 includes 5 information about pleural effusion, sub flank mass, oliguria, nausea and vomiting, and anorexia. The importance of Y2 in descending order of information is dullness and subjugation. They contain more than 95% of the information in this category. Combined with the analysis of professional knowledge, this information group roughly reflects the pathogenesis of the positive, virtual, and evil knots.

The latent variable Y3 includes 6 information about thin stools, tinnitus, night sweats, dull complexion, pale complexion, and yellow complexion. The importance of Y3 information in descending order is dull complexion, night sweats, thin stools, tinnitus, and yellow complexion. They contain more than 95% of the information in this category. Combined with the analysis of professional knowledge, this information group roughly reflects the pathogenesis of spleen and kidney deficiency.

The latent variable Y4 includes 6 information about pulse astringency, dry stool, varicose veins under the tongue, petechiae tongue, fat large tooth-marked tongue, and purple tongue. The information of importance to Y4 in descending order is purple tongue, fat large tooth-marked tongue, sublingual collateral varicose, petechiae tongue, and they contain more than 95% of the information in this category. Combined with professional knowledge analysis, this information group is based on the classification of pathological tongue picture, suggesting the pathogenesis of blood stasis internal resistance.

The article "Research on Classification of Primary Liver Cancer Syndrome Based on Data Mining Technology" was retracted in 2023. Reasons: signs of a paper mill; compromised peer review; unreliable results or conclusions.

The latent variable Y5 includes 3 information about greasy fur, yellow fur, and white fur. According to this information, the research population can be divided into 3 hidden categories. This information group is based on the classification of the tongue picture, which roughly reflects the pathogenesis of water dampness, cold, or heat.

The latent variable Y6 only has an effect on the appearance of one red tongue message, implying that it is connected to heat.

The latent variable Y7 includes information about liver palm spider nevus and lip and nail bruising. The most important information for Y7 is lip turban bruising and liver palm spider nevus. Combined with professional knowledge analysis, this information group roughly reflects the pathogenesis of blood stasis internal resistance.

The latent variable Y8 includes 5 information about pulse number, ascites, hot flashes, fever, and pale nails. The most important information for Y8 is fever and hot flashes. They contain more than 95% of information in this category. Combined with professional knowledge analysis, this information group roughly reflects the pathogenesis of liver cancer fever.

The hidden variables Y9 and Y10 are all classified based on pulse conditions. According to the four pulse conditions, Y9 can divide the research population into three hidden categories, namely, slippery pulse, stringy pulse, and weak pulse, which roughly reflects the pathogenesis of liver cancer.

The latent variable Y11 includes 5 information about fatigue, weakness of waist and knees, insomnia, frequent nocturia, and bad mouth. The importance of Y11 information in descending order is fatigue, waist and knee weakness, insomnia, and frequent nocturia. They contain more than 95% of the information in this category. Combined with professional knowledge analysis, this information group roughly reflects the pathogenesis of liver and kidney deficiency.

The latent variable Y12 includes 4 information about hand-foot-heart heat, thirst, bitter mouth, and dry mouth and throat. The importance of Y12 information in descending order is dry mouth; bitter mouth; and hot hands, feet, and heart. They contain more than 95% of the information in this category. Combined with professional knowledge analysis, this information group roughly reflects the pathogenesis of yin deficiency and internal heat.

The article "Research on Classification of Primary Liver Cancer Syndrome Based on Data Mining Technology" was retracted in 2023. Reasons: signs of a paper mill; compromised peer review; unreliable results or conclusions.

The latent variable Y13 includes 5 information about shoulder and back pain, yellow urine, hiccup and warm air, lower extremity edema, and yellowing of the body. The importance of Y13 in descending order of information is yellow urine, hiccups, yellowing of the body, and lower extremity edema. They contain more than 95% of the information in this category. Combined with the analysis of professional knowledge, this information group roughly reflects the pathogenesis of liver and gallbladder damp-heat.

Based on the above interpretation of the pathogenesis law explained by the hidden variables, we have preliminarily obtained information on liver qi stagnation syndrome, internal blood stasis syndrome, spleen and kidney deficiency syndrome, liver and kidney deficiency syndrome, and liver-gallbladder damp-heat syndrome. There are five types of syndromes that are more common in clinical practice. Next, we plan to combine the abovementioned pathogenesis analysis to carry out further analysis of some of the syndrome elements to provide data support for the development of clinically actual syndrome diagnostic criteria.

#### 4.2.2. Comprehensive Clustering of Latent Variables

Comprehensive clustering is a subsequent processing method of implicit structure data modeling. When multiple hidden variables are simultaneously related to a syndrome or syndrome elements and reflect different aspects, it is necessary to fully consider the main four-diagnosis information data contained in these hidden variables. Perform comprehensive clustering on these hidden variables to obtain a certain type of comprehensive clustering model. At the same time, the implicit structure model combines the knowledge of information theory and probability theory, and by observing the information curve, one can draw the qualitative relationship between the syndrome or syndrome elements and the main four-diagnosis information. Observation of the probability distribution can derive the quantitative relationship between the syndrome or syndrome elements and the main four-diagnosis information. This study continues to use Lantern 3.1.2 software, selects the five syndrome elements that have an important influence on the pathogenesis of primary liver cancer, namely, stagnation of qi, water dampness, blood stasis, heat, and deficiency, to optimize the combination of latent variables, comprehensive clustering, and obtain related information curves and class probability distributions.

Qi stagnation involves three hidden variables *Y*0, *Y*l, and *Y*9. A new hidden variable *Z*1 is introduced, and *Z*1 is connected with *Y*0, *Y*1, and *Y*9. After comprehensive clustering, the information curve of *Z*1 (see Figure 1) and the class probability distribution (see Table 1) are obtained. A total of 7 information are screened out by the hidden variable *Z*1, covering at least 95% of the information of air lag. The information in descending order of importance is fullness of stomach, chills, flank pain, stomach and wrist pain, dizziness, chest tightness, and fullness of abdomen. At the same time, *Z*1 divided the study population into 2 hidden categories, which were recorded as *Z*l = *s*0 and *Z*l = *s*l, and the probability of appearance was 60% and 40% respectively. When *Z*l = *s*0, the probability of each occurrence of these 7 pieces of information is relatively higher than that when *Z*l = *s*l. Therefore, it is believed that patients with *Z*l = *s*0 have symptoms of qi stagnation, and such people account for 60% of the total sample size. According to professional knowledge, we eliminated chills and dizziness, two symptoms that are weakly related to qi stagnation syndrome in TCM. Therefore, it can be considered that hypochondriac pain, stomach and wrist pain, abdominal distension, and chest tightness are the typical clinical manifestations of stagnation of qi in liver cancer, reflecting the basic pathogenesis of liver qi stagnation and liver qi invading the stomach.

The article "Research on Classification of Primary Liver Cancer Syndrome Based on Data Mining Technology" was retracted in 2023. Reasons: signs of a paper mill; compromised peer review; unreliable results or conclusions.

Water wetness involves the three hidden variables, *Y*5, *Y*9, and *Y*13. A new hidden variable *Z*2 is introduced, and *Z*2 is connected with *Y*5, *Y*9, and *Y*13. After comprehensive clustering, the information curve of Z1 (see Figure 2) and the class probability distribution (see Table 2) are obtained. The hidden variable *Z*2 has screened out 4 pieces of information, covering at least 95% of the information about water wetness. The information in descending order of importance is stringed pulse, greasy moss, slippery pulse, and yellow urine. At the same time, *Z*2 divides the research population into 2 hidden categories, which are, respectively, marked as *Z*2 = *s*0, *Z*2 = *s*l, and the probability of appearance is 28% and 72%, respectively. When *Z*2 = *s*0, the probability of each of these 4 information appearing is relatively relative. When *Z*2 = *s*l is higher than *Z*2 = *s*1, it is considered that *Z*2 = *s*0 patients have watery symptoms, and such people account for 28% of the total sample size. Therefore, it can be considered that yellow urine, greasy moss, and slippery pulse are typical clinical manifestations of water dampness syndrome of liver cancer which is shown in Table 2.

Blood stasis involves five hidden variables, *Y*0, *Y*2, *Y*4, *Y*7, and *Y*9. A new hidden variable *Z*3 is introduced, and *Z*3 is connected with *Y*0, *Y*2, *Y*4, *Y*7, and *Y*9. After comprehensive clustering, the information curve of *Z*3 (See Figure 3) and the class probability distribution are obtained (see Table 3). The hidden variable *Z*3 has screened out 6 information, covering at least 95% of the blood stasis information. The information in descending order of importance is pulse strings, lip and nail bruising, liver palm spider nevi, purple tongue, slippery pulse, and fat and large teeth marks on the tongue. At the same time, *Z*3 divides the population of this study into two hidden categories, denoted as *Z*3 = *s*0 and *Z*3 = *s*1, respectively, with the probability of appearance being 30% and 70%, respectively. When *Z*3 = *s*0, the probability of each of these 6 messages is relatively higher than that of *Z*3 = sl. Therefore, it is believed that patients with *Z*3 = *s*0 have symptoms of blood stasis, and such people account for 30% of the total sample size. According to professional knowledge, the two symptoms of slippery pulse, fat tooth marks and tongue are eliminated. Therefore, it can be considered that lip and nail bruising, liver palm spider nevus, tongue purple, pulse string are the typical clinical manifestations of liver cancer with blood stasis syndrome.

The article "Research on Classification of Primary Liver Cancer Syndrome Based on Data Mining Technology" was retracted in 2023. Reasons: signs of a paper mill; compromised peer review; unreliable results or conclusions.

There is a hot, involving three hidden variables Y8, Y12, and Y13. Introduce a new hidden variable Z4 and it with Y8, Y12, and Y13. After comprehensive clustering, we have obtained the information curve of Z4 (see Figure 4) and class probability distribution (see Table 4). Hidden variable *Z*4 screened out 5 pieces of information, covering at least 95% of the information with heat. The information in descending order of importance is dry mouth; bitter mouth; yellow urine; hot hands, feet; and thirst. At the same time, *Z*4 divides the study population into 2 hidden categories, which are, respectively, denoted as *Z*4 = *s*0 and *Z*4 = *s*1, and the probability of occurrence is 47% and 53%, respectively. When *Z*4 = *s*0, the probability of each of these five messages appearing is relatively higher than when *Z*4 = *s*l. Therefore, it is believed that patients with *Z*4 = *s*0 have fever syndromes, and this group of people accounted for 47% of the total sample size. Therefore, it can be considered that dry mouth; thirst; bitter mouth; warm hands, feet, heart; and yellow urine are typical clinical manifestations of liver cancer fever.

Positive and imaginary variables involve five hidden variables Y2, Y3, Y10, Y11, and Y12, and we introduce a new hidden variable Z5 and connect Z5 with Y2, Y3, Y10, Y11, and Y12. After comprehensive clustering, the hidden variable Z5 will be used. The population is divided into 3 hidden categories. According to professional knowledge, this category can be considered to include two subcategories of spleen and kidney yang deficiency and liver and kidney deficiency. Among them, *Y*2, *Y*3, *Y*10 are related to spleen and kidney deficiency, and *Y*10, *Y*11, and *Y*12 are related to liver and kidney deficiency. Furthermore, comprehensive clustering is performed on these variables, and the latent variables Z5a and Z5b are introduced, respectively.

The article "Research on Classification of Primary Liver Cancer Syndrome Based on Data Mining Technology" was retracted in 2023. Reasons: signs of a paper mill; compromised peer review; unreliable results or conclusions.

Combining the information curve (see Figure 5) and the class probability distribution (see Table 5), *Z*5a has screened out 5 pieces of information, covering at least 95% of the information on the deficiency of both spleen and kidney, in descending order of importance. The small messages are, in order, thin pulse, dull complexion, thin stool, weak pulse, and tinnitus. At the same time, *Z*5a divides the research population into 2 hidden categories, which are, respectively, denoted as *Z*5a = *s*0 and *Z*5a = *s*l. The probability of occurrence is 69% and 31%, respectively. However, when *Z*5a = *s*0, the probability of each of these 5 messages appearing is relatively higher than when *Z*5a = *s*1, so it is believed that patients with *Z*5a = *s*0 have syndromes of deficiency of both spleen and kidney. And, this group of people accounted for 69% of the total sample size. Therefore, it can be considered that dull complexion, tinnitus, loose stools, and weak pulse are the typical clinical manifestations of liver cancer with deficiency of both spleen and kidney.

Combining the information curve (see Figure 6) and the class probability distribution (see Table 6), *Z*5b has screened a total of 6 information, covering at least 95% of the information on liver and kidney deficiency. According to the information in descending order of importance, they are dry mouth and throat, fatigue, waist and knees, pain in the mouth, insomnia, and frequent nocturia. At the same time, *Z*5b divides the research population into 2 hidden categories, which are, respectively, denoted as *Z*5b = *s*0 and *Z*5b = *s*1, and the probability of emergence is 31% and 69%, respectively. When *Z*5b = *s*0, the probability of each of these 6 messages is relatively higher than when *Z*5b = *s*1, so it is believed that patients with *Z*5b = *s*0 have symptoms of liver and kidney deficiency. And, this group of people accounted for 31% of the total sample size. According to professional knowledge, the symptom of bitter mouth can be eliminated by comparing dry mouth and throat. Therefore, it can be considered that dry mouth, dryness of the throat, fatigue, weakness of waist and knees, insomnia, and frequent nocturia are the typical clinical manifestations of liver cancer and liver and kidney insufficiency.

The article "Research on Classification of Primary Liver Cancer Syndrome Based on Data Mining Technology" was retracted in 2023. Reasons: signs of a paper mill; compromised peer review; unreliable results or conclusions.

In summary, based on the analysis of the hidden structure model, this study explored six clinically common symptoms of primary liver cancer: qi stagnation syndrome, water dampness syndrome, blood stasis syndrome, heat syndrome, spleen and kidney deficiency syndrome, and liver and kidney deficiency syndrome. The corresponding relationship between the syndromes and the four-diagnosis information of TCM is specifically as follows:

  Qi stagnation syndrome, typical clinical manifestations include hypochondriac pain, stomach pain, abdominal distension, and chest tightness
  Water dampness syndrome, typical clinical manifestations include yellow urine, greasy fur, and slippery pulse
  Blood stasis syndrome, typical clinical manifestations include lip and nail bruising, liver palm spider nevus, purple tongue, pulse string
  Heat syndrome, typical clinical manifestations include dry mouth and throat; thirst; bitter mouth; warm hands, feet, and heart; and yellow urine
  The syndrome of spleen and kidney deficiency, typical clinical manifestations include dull complexion, tinnitus, stool, and weak pulse
  Insufficiency of liver and kidney, typical clinical manifestations include dry mouth and throat, fatigue, weakness of waist and knees, insomnia, and frequent nocturia

### 4.3. The Results of Factor Analysis and Joint Cluster Analysis

Factor analysis is an unsupervised data mining technique that analyzes the role of factors hidden behind the surface phenomenon of the data. It reduces multivariate data into a few representative “factors” through “dimensionality reduction and order upgrade.” Use these “factors” to summarize and explain the largest number of observations to reveal the nature of the relationship between variables. The 57 four-diagnosis information data of Chinese medicine in this study can be regarded as 57 directly observable and relevant variable data.

Through factor analysis, this study made a preliminary classification of the four-diagnosis information of inpatients with liver cancer. In order to deeply explore the connotation of syndromes of liver cancer, it is necessary to classify similar factors according to the pathogenesis of traditional Chinese medicine and establish a factor loading matrix of a certain category. This study is based on the abovementioned syndrome clustering research results. Combining the basic pathogenesis of liver cancer in traditional Chinese medicine, optimize the combination of factors and comprehensively evaluate them. Obtain the relevant load matrix, and screen the syndrome elements in each classification.

The article "Research on Classification of Primary Liver Cancer Syndrome Based on Data Mining Technology" was retracted in 2023. Reasons: signs of a paper mill; compromised peer review; unreliable results or conclusions.

Firstly, interpret the pathogenesis rules suggested by the main four-diagnosis information contained in the 23 factors.

  Factor 1: it mainly suggests the pathogenesis of liver and kidney deficiency
  Factor 2: it is a classification based on pathological tongue picture, which mainly indicates the pathogenesis of blood stasis
  Factor 3: it is still based on the classification of tongue picture, which mainly indicates the pathogenesis of water dampness
  Factor 4: the disease is located in the spleen and stomach, which is a manifestation of spleen and stomach disharmony, indicating qi deficiency and qi stagnation
  Factor 5: the disease is located in the liver and stomach, which mainly indicates the pathogenesis of liver stagnation and qi stagnation
  Factor 6: all are related to fever, mainly indicating fever
  Factor 7: the location of the disease is related to the accumulation of water and dampness
  Factor 8: the classification is based on the pulse condition, and the pathogenesis has two ends of deficiency and excess
  Factor 9: it may indicate heat
  Factor 10: it is based on the classification of tongue coating, which mainly indicates the pathogenesis of damp heat
  Factor 11: it mainly indicates stagnation and heat
  Factor 12: it reflects the pathogenesis of deficiency of both qi and blood
  Factor 13: it may not raise blood stasis
  Factor 14: it may be related to qi stagnation and dampness resistance, mainly indicating water dampness and qi stagnation
  Factor 15: it mainly suggests qi stagnation
  Factor 16: unclear pathogenesis
  Factor 17: It mainly suggests the pathogenesis of blood stasis
  Factor 18: it roughly reflects the pathogenesis of the spleen and kidney deficiency
  Factor 19: it is the manifestation of liver and gallbladder damp-heat pathogenesis
  Factor 20: it may be related to water humidity

Based on factor analysis combined with cluster analysis, this study explored six primary liver cancer syndromes: liver qi stagnation syndrome, spleen deficiency and dampness syndrome, liver blood stasis syndrome, liver and gallbladder damp-heat syndrome, spleen and kidney deficiency syndrome, and liver and kidney deficiency syndrome. Correspondence between common clinical syndromes and the information of the four diagnoses of TCM, specifically:

  Liver stagnation and qi stagnation syndrome, typical clinical manifestations include hypochondriac pain, stomach pain, nausea and vomiting, heavy head and sleepiness, emotional depression, and red tongue
  Spleen deficiency and dampness syndrome, typical clinical manifestations include dull complexion, abdominal distension, heavy head and body, pleural fluid, stool, and white fur
  Liver blood stasis syndrome, typical clinical manifestations include chest pain, liver palm spider mole, purple tongue with petechiae, sublingual varicose veins, and astringent pulse
  Liver and gallbladder damp-heat syndrome, typical clinical manifestations include fever, dry stool, yellow and greasy fur
  The syndrome of spleen and kidney deficiency, typical clinical manifestations include pale and dull complexion, tinnitus, and oliguria
  Insufficiency of liver and kidney, typical clinical manifestations include dry mouth and throat; thirst; fatigue; warm hands, feet, and heart; frequent nocturia; and weak pulse

The article "Research on Classification of Primary Liver Cancer Syndrome Based on Data Mining Technology" was retracted in 2023. Reasons: signs of a paper mill; compromised peer review; unreliable results or conclusions.

## 5. Conclusion

This study used systematic clustering analysis to find that the clinical symptoms of liver cancer were qi stagnation, stagnation of qi and blood stasis, mutual accumulation of dampness and blood stasis, dysfunction and blood stasis, flaming heat toxins, liver and gallbladder dampness and heat, liver and kidney deficiency, and yang deficiency of the spleen and kidney. However, due to hierarchical clustering, each piece of information will only be simply classified into a specific category. When discussing the clustering results based on professional knowledge, some deviations will inevitably occur. Liver and gallbladder dampness and heat, and liver and kidney deficiency were grouped into the same syndrome category; this is not entirely in line with clinical reality. Then, using the hidden structure model through preliminary clustering, we obtained 5 types of clinical common syndromes of primary liver cancer with liver qi stagnation syndrome, blood stasis syndrome, spleen and kidney deficiency syndrome, liver and kidney deficiency syndrome, and liver-gallbladder damp-heat syndrome. It also interprets the syndrome elements from the perspective of pathogenesis, and further optimizes the combination of similar syndrome elements through comprehensive clustering. Discuss the common syndromes and the typical clinical manifestations of six types of liver cancer with qi stagnation syndrome, water dampness syndrome, blood stasis syndrome, heat syndrome, spleen and kidney deficiency syndrome, and liver and kidney deficiency syndrome, respectively. Specifically, they are qi stagnation syndrome, water dampness syndrome, blood stasis syndrome, heat syndrome, spleen and kidney deficiency syndrome and liver and kidney deficiency syndrome. Finally, using factor analysis combined with common factor clustering, information on seven types of liver cancer were obtained: liver stagnation and qi stagnation, liver stagnation and qi stagnation to transform fire, stagnation of qi and blood stasis, liver and blood stasis, spleen deficiency and dampness, liver and kidney deficiency, and spleen and kidney deficiency. At the same time, with the help of pathogenesis analysis, the syndrome elements were classified and interpreted, and the factor loading matrix was established to comprehensively evaluate the syndrome of liver qi stagnation, spleen deficiency and dampness syndrome, liver and blood stasis syndrome, liver and gallbladder damp-heat syndrome, spleen and kidney deficiency syndrome, and insufficiency of liver and kidney. These are the 6 common syndromes of liver cancer and their typical clinical manifestations.

The article "Research on Classification of Primary Liver Cancer Syndrome Based on Data Mining Technology" was retracted in 2023. Reasons: signs of a paper mill; compromised peer review; unreliable results or conclusions.

## Figures and Tables

**Figure 1:** Information curve graph of hidden variable *Z*1.

**Figure 2:** Information curve graph of hidden variable *Z*2.

**Figure 3:** Information curve graph of hidden variable *Z*3.

**Figure 4:** Information curve graph of hidden variable *Z*4.

**Figure 5:** Information curve graph of hidden variable *Z*5a.

**Figure 6:** Information curve graph of hidden variable *Z*5b.

**Table 1:** Class probability distribution table of implicit probability *Z*1.

Item	*Z*1 = *s*0 (%)	*Z*1 = *s*1 (%)
Gastric cavity swelling	87	60
Stomach cold	92	52
Flank rib pain	70	80
Gastric cavity pain	98	31
Dizziness	90	45
Chest tightness	96	33
Bloating	91	25

**Table 2:** Class probability distribution table of implicit probability *Z*2.

Item	*Z*2 = *s*0 (%)	*Z*2 = *s*1 (%)
Pulse string	92	78
Greasy fur	81	72
Slippery pulse	97	28
Yellow urine	51	34

**Table 3:** Class probability distribution table of implicit probability *Z*3.

Item	*Z*3 = *s*0 (%)	*Z*3 = *s*1 (%)
Pulse string	86	78
Labial nail cyan	96	55
Liver palm spider nevus	97	29
Purple tongue	79	65
Slippery pulse	97	29
Fat tooth mark tongue	79	51

**Table 4:** Class probability distribution table of implicit probability *Z*4.

Item	*Z*4 = *s*0 (%)	*Z*4 = *s*1 (%)
Dry mouth	89	76
Bitter mouth	93	62
Yellow urine	88	60
Hot hands, feet, and heart	97	32
Thirsty	100	20

**Table 5:** Class probability distribution table of implicit probability *Z*5.

Item	*Z*5a = *s*0 (%)	*Z*5a = *s*1 (%)
Thin pulse	83	79
Dull complexion	58	86
Loose stools	91	39
Weak pulse	93	37
Tinnitus	97	28

**Table 6:** Class probability distribution table of implicit probability *Z*5b.

Item	*Z*5b = *s*0 (%)	*Z*5b = *s*1 (%)
Dry mouth	95	41
Fatigue	88	29
Sore waist and knees	97	59
Bitter mouth	93	57
Insomnia	94	62
Frequent nocturia	95	63

## Data Availability

The datasets used and analyzed during the current study are available from the corresponding author upon reasonable request.
